# Long Noncoding RNA CASC2 Facilitated Wound Healing through miRNA-155/HIF-1*α* in Diabetic Foot Ulcers

**DOI:** 10.1155/2022/6291497

**Published:** 2022-06-24

**Authors:** Minjie He, Liang Tu, Ruo Shu, Qi Meng, Sicheng Du, Zhao Xu, Shaoyun Wang

**Affiliations:** ^1^Geriatric Department, First Affiliated Hospital of Kunming Medical University, 295 Xichang Road, Kunming 650000, Yunnan, China; ^2^Medical Experimental Center, The First Affiliated Hospital of Chongqing Medical and Pharmaceutical College (The 6th People Hospital of Chongqing), 301 Nancheng Road, Chongqing 400060, China; ^3^Department of Gastrointestinal Surgery, First Affiliated Hospital of Kunming Medical University, 295 Xichang Road, Kunming 650000, Yunnan, China; ^4^Department of General Medicine, First Affiliated Hospital of Kunming Medical University, 295 Xichang Road, Kunming 650000, Yunnan, China; ^5^Endocrinology Department, First Affiliated Hospital of Kunming Medical University, 295 Xichang Road, Kunming 650000, Yunnan, China; ^6^Department of Orthopedics, First Affiliated Hospital of Kunming Medical University, 295 Xichang Road, Kunming 650000, Yunnan, China

## Abstract

Diabetic foot ulcers (DFU) are among the serious complications which are closely linked to diabetes mellitus. However, there is still a lack of accurate and effective standard prevention and treatment programs for DFU. In this manuscript, we have investigated the function of lncRNA cancer susceptibility candidate 2 (CASC2)/miR-155/hypoxia-inducible factor 1-alpha (HIF-1*α*) in the wound healing of DFU. We have analyzed lncRNA CASC2`s expression in the marginal tissues of ulcers in patients and mice with DFU. Additionally, the interaction relationship and mechanism between lncRNA CASC2, miR-155, and HIF-1*α* were determined, which proved the effects of lncRNA CASC2/miR-155/HIF-1*α* on fibroblasts apoptosis, proliferation, and migration. According to our study, the lncRNA CASC2's expression was low in the tissues of ulcers of DFU mice and patients. lncRNA CASC2's overexpression promoted fibroblasts migration, proliferation, and inhibited apoptosis and was beneficial for the healing of wounds, preferably in the DFU mice. In addition, lncRNA CASC2 directly targets miR-155 and HIF-1*α* functions as miR-155's target gene. Overexpression of miR-155 abrogated the function of lncRNA CASC2. Similarly, HIF-1*α*'s inhibition has reversed the effect of miR-155 downregulation on fibroblasts. In general, overexpression of lncRNA CASC2 facilitated wound healing through miR-155/HIF-1*α* in DFU.

## 1. Introduction

Throughout the world, diabetes mellitus (DM) is assumed as a challenging disease, i.e., chronic metabolic, and its prevalence is increasing constantly with time [1]. Diabetic foot ulcer (DFU) is a serious and extended complication of DM, which is difficult to treat and serves as a considerable medical care burden. DFU is a foot infection, ulcer, and deep-tissue destruction caused by long-term hyperglycemia that causes abnormalities in the distal peripheral nerves of the lower limbs and various degrees of microvascular disease [2–4]. Its characterization is closely linked to impair healing of wounds, particularly in the lower extremities. Due to repeated infections of the wound, poor local blood supply, and uneven force on the feet, the wound is prolonged and difficult to heal; therefore, the treatment effect is often poor. A quarter of patients with diabetes are at an increased risk of foot injury due to diabetic neuropathy and vascular disease. The rate of new foot lesions in diabetics is 3% to 7% per year. After foot injury heals, the risk of secondary ulcers increases gradually, between 30% and 100%, depending on the quality of follow-up care. As with other types of amputation in the past, diabetics must be considered a high-risk group for amputation, requiring careful and planned monitoring and care. More than 20,000 diabetics in Germany each year have foot lesions that eventually require amputation. The mortality rate after amputation is approximately 20%. Within three years of amputation, 50% of survivors still need to have the contralateral lower limb amputated. The 5-year survival rate after amputation is low, about 25% [2–4].

Long noncoding RNA (lncRNA) is a special type of the original RNA molecule where the transcript is particularly longer than 200 nt and does not encode any proteins [5, 6]. The expression of lncRNA is regulated by the up-growth and is specific in tissues and cells. lncRNA Cancer Susceptibility Candidate 2 (CASC2) was originally discovered in the endometrial cancer (EC) study and is located on human chromosome 10q26 [7]. There is evolutionary conservation in sequence and highly homologous sequences between species, which is the potential tumor suppressor gene. Previous studies [8–10] have found that CASC2 is involved in the pathological process of regulating diabetes and its complications.

lncRNA functions as a competitive endogenous RNA (ceRNA) to interact with microRNA (miRNA) and take part to regulate the target gene's expression [11]. On the contrary, miRNA regulates lncRNA to perform biological functions via RNA-induced silencing complex (RISC) [12, 13]. LncRNA CASC2 utilized the function of suppressive tumor in the cancer of the pancreatic by using the miR-24/MUC6 axis, which is assumed as one of the prominent targets in the therapy of pancreatic [14]. In addition, lncRNA CASC2 is used for the reduction of the process and degree of apoptosis, fibrosis, and inflammation, particularly in the models of diabetic nephropathic where miR-144/SOCS2 axis is regulated properly [15]. The regulation of miRNA on target genes is manifested at the level of posttranscriptional, and target genes expression is downregulated through the inhibition process of target gene mRNA translation. For example, miR-155 inhibitors can reduce the oxidative stress-related molecules accumulation and prevent damage to mitochondrial and cardiomyocyte apoptosis through the increasing pathway of nuclear factor erythroid 2-related factor 2/heme oxygenase-1 (Nrf2/HO-1) signaling, thereby improving diabetic myocardial fibrosis [16]. More importantly, miR-155 also plays a significant role in diabetic foot ulcers. MiR-155 worsened the function of endothelial progenitor cells (EPC) persuaded via high glucose by downregulating PTCH1 [17]. Inhibition of microRNA-155 restores the expression of fibroblast growth factor 7 (FGF7) in diabetic skin and reduces wound inflammation, increases epithelial formation, and therefore accelerates wound closure [18]. These suggest that downregulation of miR-155 promoted the healing of wounds in rats (DFU).

Hypoxia-inducible factor-1*α* (HIF-1*α*), as an endogenous protective molecule, contributes to the cellular process of the healing of wounds [19] such as activating angiogenic factors to stimulate angiogenesis [20] and promoting EPC recruitment to the wound site [21]. Some studies [22–24] have found that miR-155 regulates HIF-1*α* in a targeted manner. Therefore, this study investigated the role of lncRNA CASC2/miR-155 /HIF-1*α* in DFU wound healing, hoping to provide a new idea for DFU treatment.

The remaining portions or sections of this paper are arranged as follows.

In the following section, the proposed methodology, preferably from sample selection to proper experimental setup and its realization, is explained with sufficient details along with basic requirements. In Section 3, numerous experimental results along with sufficient explanations are presented. For understandability, these results were provided in both textual and graphical formats. Finally, concluding remarks are given along with future directives.

## 2. Methods

### 2.1. Ethical Statement

Twenty-five samples were gathered from the ulcer edge tissue samples of DFU patients and twenty-five samples from the distal end tissue samples of orthopedic amputation patients without diabetic trauma from June 2021 to June 2022. It is important to note that each patient, who participated in the proposed study, has signed a written consent letter where proper information was provided about this study. Furthermore, this experiment was approved through the Ethics Committee which is formed in the First Affiliated Hospital of Kunming Medical University. These experiments were carried out by observing strict compliance which was according to the Herki Declaration. Animal experiments, which were performed, were permitted by the Use Committee and Animal Care of the Kunming Medical University and comply with the procedure and guidelines for the use and care of animals. These guidelines were set by the National Institutes of Health (NIH).

### 2.2. Cell Isolation, Culture, and Transfect

We have taken a skin (preferably with full-thickness) graft (1.0 cm^2^) from the ulcer marginal tissue of a DFU patient and placed it in a DMEM medium containing 10% fetal bovine serum (FBS, Gibco, NY, USA). Wash with phosphate buffer saline (PBS, Bio-Channel, Nanjing, China) containing 100 U/mL penicillin-streptomycin (Thermofisher Scientific, MA, USA) and incubate at a temperature of 37°C and CO_2_ of 5% in DMEM medium containing FBS 10%. When the cells grow to 80%–90%, they are passaged. Cells from 35 generations were used in subsequent experiments. A Lipofectamine 3000 kit, which is collected from Invitrogen, CA, USA, was used for the transfection of cells and was carried out according to the manufacturer's instructions.

### 2.3. Reverse Transcription Quantitative Polymerase Chain Reaction (RT-qPCR)

The TRIzol reagent (Leagene, Beijing, China) extracts total RNA from cell and tissue samples. The RNA is reverse transcribed into cDNA according to the reverse transcription kit (Takara, Tokyo, Japan). cDNA was used as a template, SYBR Green PCR Master Mix (Thermofisher Scientific, MA, USA) was used for RT-qPCR reaction, GAPDH and U6 were utilized as internal reference genes. Relative expression of target gene mRNA in each sample was calculated according to the Ct value of PCR reaction signal intensity and the change of mRNA level of expression was computed by the mechanism of 2^−ΔΔCt^. The sequences are CASC2 F; 5′-GCACATTGGACGGTGTTTCC-3′, R:5′-CCCAGTCCTTCACAGGTCAC-3′; miR-155F; 5′-ACACTCCAGCTGGTTAATGCTAATCGTGAT′, R; 5′- TTAATGCTAATCGTGATAGGGGT-3′; HIF-1*α* F; 5′- GGCAACCTTGGATTGGATGG-3′, R: 3′-TCTCCGTCCCTCAACCTCTC-5'; GAPDH F:5′-AATCCCATCACCATCTTCCA-3′, R; 5′- TGGACTCCACGACGTACTCA-3′; U6 F: 5′-TCCGATCG TGAAGCGTTC-3′, R; 5′ -GTGCAGGGTCCGAGGT-3′.

### 2.4. Western Blot (WB)

The RIPA lysis solution (Beyotime, Beijing, China) was utilized to extract tissue and cell proteins, whereas the concentration of the protein was found through the bicinchoninic acid (BCA, Ricky, Shanghai, China). After separation by SDS-PAGE electrophoresis (Aowei, Shanghai, China), transfer to PVDF membrane, then block with 5% skim milk, add primary antibody HIF-1*α*, VEGF, collagen-I (Col-I), and GAPDH (1 : 1000, Cell Signaling Technology, MA, USA), incubate overnight at 4°C, and incubate the secondary antibody (CST) at 37°C for 1 h. Use the ECL Plus (Fluorescence, Beijing, China) to develop color and the gel imaging system (Image J) to scan and analyze the protein bands.

### 2.5. Flow Cytometry

Apoptosis of cells was determined through the manual instructions which were provided by the cell apoptosis detection kit (Sigma-Aldrich, MO, USA). Annexin V-FITC, propidium iodide (PI), and buffer are mixed and used to incubate the cells, then resuspend the cells in the buffer, and detect them with a flow analyzer.

### 2.6. Wound Healing

Cells are stored into a plate of six-wells. When the cells are almost confluent, scratch the well plate vertically with a 10 *μ*L pipette tip and culture in a serum-free medium (Gibco). Observe the cell migration distance at 0 h and 24 h.

### 2.7. Dual-Luciferase Reporter

The binding region of CASC2/HIF-1*α* and miR-155 was determined by the Starbase database. Construct a recombinant plasmid linked to the pGL3 vector (Promega, WI, USA): CASC2 wild-type (pGL3-CASC2-wt), CASC2 mutant (pGL3-CASC2-mut), HIF-1*α* wild-type (pGL3-HIF-1*α*-wt), and HIF-1*α* mutant (pGL3-HIF-1*α*-mut). The recombinant plasmid was cotransfected with miR-155 mimics (Aibiqi, Shanghai, China) or negative control (NC, Aibiqi). After 24 hours, the cells were collected to determine the intracellular luciferase activity.

### 2.8. MTT Assay

In brief, add 5 × 10^3^ cells to a plate of ninety-six (96) wells, and the incubation process is performed at a temperature level of 37°C, 5% CO_2_ for 24 hours. Then, the MTT solution (Medchem Express, NJ, USA) was added to the culture medium for 4 hours, and dimethyl sulfoxide was added and shaken for 10 minutes to remove crystals, whereas absorbance was calculated at 490 nm.

### 2.9. Construction of DFU Mice Model

The ICR male mice, whose ages were between six to eight weeks, was bought from the Animal Center of Kunming University of Science and Technology. All mice were kept in an environment with a temperature of 22 ± 1°C, a humidity of 50 ± 10%, and a 12 h day and night alternate. Intraperitoneal injection of streptozotocin (STZ, 50 mg/kg, InvivoChem, CA, USA), after 72 h, the blood glucose of the mice was measured, and the mice showed continuous blood glucose ≥16.7 mmol/L as diabetic mice. After the diabetic mice were successfully constructed, the mice were anesthetized and the skin of the mice feet (4 cm^2^) was removed and injected with the CASC2 overexpression plasmid packaged with lentivirus or PBS for intervention. Images of mouse foot injury were collected on day 3, day 8, and day 16.

### 2.10. Statistical Analysis

We have expressed the experimental results, which are collected through the experimental setup and procedures, in the form of standard deviation (SD) and mean ±. Furthermore, GraphPad Prism 5.0 software, which is a dedicated software designed for statistics, was utilized to examine and analyze the collected experimental data values. To compare data values and performance of these two groups, we have utilized the Student's *t*-test along with a one-way analysis of variance, preferably for two (02) or more groups. From this analysis, we have observed a statistically significant difference, that is, *p* < 0.05.

## 3. Experimental Results and Observations

### 3.1. The Levels of LncRNA CASC2 and Mir-155 in DFU Patients

We have detected various levels of expression of the lncRNA miR-155 and CASC2 in the ulcer marginal skin of 25 DFU patients and the normal foot tissues of 25 healthy individuals (control group). The results showed that lncRNA CASC2 was lowly expressed in the ulcer marginal tissues of DFU patients compared with the control group (Figure 1(a)). While miR-155 is highly expressed in the ulcer marginal tissues of DFU patients than in normal foot tissues (Figure 1(b)). Moreover, the expression levels of lncRNA CASC2 and miR-155 are negatively correlated in the marginal tissues of foot ulcers in patients with DFU (Figure 1(c)).

### 3.2. LncRNA CASC2 Facilitated Wound Healing In Vitro and In Vivo

To explore the role of lncRNA CASC2 in the healing of ulcers in DFU patients, we isolated fibroblasts from ulcer marginal tissues and transfected them with the lncRNA CASC2 overexpression vector and empty vector as a negative control (NC). The expression of lncRNA CASC2 increased after transfection with lncRNA CASC2 (Figure 2(a)). Flow cytometry demonstrated that increased expression of lncRNA CASC2 reduced fibroblast apoptosis (Figures 2(b) and 2(c)). Subsequently, transfection of lncRNA CASC2 overexpression vector promoted the migration of fibroblasts (Figure 2(d)). While we analyzed the proliferation activity of fibroblasts, the result showed that the cells in the CASC2 group proliferated more actively (Figure 2(e)). In addition, lncRNA CASC2 promoted wound healing in DFU mice (Figure 2(f)). Compared with the DFU mice, the expression of lncRNA CASC2 and the protein levels of HIF-1*α*, VEGF, and Col-I increased significantly in DFU + CASC2 mice (Figures 2(g) and 2(h)). The results indicated that overexpression of lncRNA CASC2 promoted wound healing in DFU cells and mice.

### 3.3. Targeted Relationship between LncRNA CASC2 and MiR-155

Therefore, we investigated the relationship between lncRNA CASC2 and miR-155, which have a binding site (Figure 3(a)). Meanwhile, the dual-luciferase reporter gene verified that the fluorescence activity was significantly decreased when cotransfected miR-155 mimics and lncRNA CASC2-wt, while the fluorescence activity remains unchanged when cotransfected miR-155 mimics and lncRNA CASC2-mut (Figure 3(b)). The result of RT-qPCR displayed that miR-155 mimics result in reduced levels of expression lncRNA CASC2, and miR-155 inhibitor results in elevated levels of expression lncRNA CASC2 (Figure 3(b)). These data suggested that lncRNA CASC2 binds to miR-155 and lncRNA CASC2 directly targets miR-155.

### 3.4. LncRNA CASC2 Regulates Cell Apoptosis, Proliferation, and Migration through Targeting MiR-155

To further determine whether lncRNA CASC2 affects the behavior of fibroblasts through miR-155, analyze cell apoptosis, proliferation, and migration after overexpression of lncRNA CASC2 and miR-155. RT-qPCR results showed that lncRNA CASC2's expression increased dramatically after lncRNA CASC2's overexpression, but the lncRNA CASC2's expression decreased after lncRNA CASC2's overexpression and miR-155 (Figure 4(a)). MiR-155's overexpression abolished the cell apoptosis inhibitory effect of increased lncRNA CASC2 (Figure 4(b)). Similarly, the increase of miR-155 abolished the promotion effect of SNHG3 addition on cell proliferation and migration (Figures 4(c) and 4(d)). We have described that the levels of expressions of vascular endothelial growth factor (VEGF), HIF-1*α*, collagen-I (Col-I), overexpression of lncRNA CASC2 facilitated the increase of HIF-1*α*, VEGF, and Col-I levels but blocked by overexpression of miR-155 (Figure 4(e)). These data indicated that lncRNA CASC2 regulates cell apoptosis, proliferation, and migration by directly targeting miR-155 in fibroblasts derived from DFU patients.

### 3.5. HIF-1*α* Functions as a Target of MiR-155

Bioinformatics analysis of the Starbase database predicts that HIF-1*α* is the target of miR-155, and Figure 5(a) is its binding site. Next, the dual-luciferase reporter gene experiment proved that miR-155 mimics reduced the activity of HIF-1*α*-wt, while the activity of HIF-1*α*-mut was unaffected (Figure 5(b)). Furthermore, we also found that the increase of miR-155 significantly inhibited the expression of HIF-1*α* mRNA and protein, and the inhibition of miR-155 increased the level of HIF-1*α* mRNA and protein (Figures 5(c) and 5(d)). These results clarified that HIF-1*α* is the target miR-155 gene.

### 3.6. MiR-155 Affected Fibroblast Apoptosis, Migration, and Proliferation via HIF-1*α*

To identify the downstream mechanism of miR-155, fibroblasts were treated with si-miR-155 and si-HIF-1*α*. Treatment of si-miR-155 downregulates the expression of miR-155 and upregulates the expression of HIF-1*α*. Treatment of si-miR-155 and si-HIF-1*α* has increased miR-155 expression and decreased HIF-1*α* as shown in Figures 6(a) and 6(b). Deleting miR-155 inhibits fibroblast apoptosis and promotes proliferationand migration, but these effects were recovered by si-HIF-1*α* (Figures 6(c)–6(e)). Additionally, the expression levels of HIF-1*α*, VEGF, and Col-I protein increased after miR-155 was knockdown, whereas knockdown of HIF-1*α* affected the expression of these proteins.

## 4. Discussion

Long-term diabetes causes ischemic, neurological, and neuroischemic lesions of the foot [25], leading to infections of different lengths, and severe cases face the risk of amputation [26]. The current treatment of DFU was maintained unsatisfactory. In this study, we investigated the role of lncRNA CASC2 in the development of DFU and found that lncRNA CASC2 directly targeted miR-155 to regulate the expression of HIF-1*α*. Consequently, overexpression of lncRNA CASC2 promoted fibroblast proliferation, migration, and inhibits apoptosis through miR-155/HIF-1*α*, which indicated that it is facilitated to wound healing with DFU (Figure 2).

Our research showed the lower level of lncRNA CASC2 in the ulcer marginal tissues of DFU patients and mice and the higher level of miR-155 in DFU patients. LncRNA CASC2 is a newly identified lncRNA that has been found to have an inhibitory effect in several types of tumors [27–29]. Previous studies by Zhang et al. revealed that the expression of lncRNA CASC2 is reduced in diabetic patients and high glucose (HG) induced cells, upregulation of CASC2 inhibits HG-induced HMC proliferation, extracellular matrix accumulation (ECM) accumulation, and oxidative stress [30]. MiR-155 has been emphasized to play an indispensable role in atherosclerosis [31], allergic asthma [32], and malignant tumors [33, 34]. In addition, miR-155 inhibition can reduce acute wound inflammation and promote wound healing in diabetic rats [35], which is consistent with our results of silencing miR-155 to inhibit fibroblast apoptosis and promote proliferation and migration (Figure 4).

This study confirmed that lncRNA CASC2 directly targets miR-155 to perform biological functions in DFU-derived fibroblasts. Recently some findings prove the influence of interaction between miR-155 and lncRNA CASC2 on several pathological processes (Figures 3 and 4). For instance, the overexpression of CASC2 inhibits the invasion and proliferation of NK-92 cells and promotes apoptosis by targeting miR-155-5p, and upregulating the expression of APC was proved by zheng et. al [36]. Wang et al. [37] indicated that one of the potential targets is CASC2 of sepsis-induced acute kidney injury (AKI) by inhibiting the NF-*κ*B and miR-155 pathways mediated inflammation.

Furthermore, we have determined that HIF-1*α* is the target gene of miR-155, knocking down HIF-1*α* abolishes the effect of miR-155 silencing on cell apoptosis, proliferation, and migration (Figures 5 and 6). The stability of HIF-1*α* is essential to the process of diabetic wound healing and accelerates wound repair through HIF-1*α* mediation [38, 39]. Zhang et al. [40]. found that human umbilical cord mesenchymal stem cells produced exosomes promote angiogenesis through HIF-1*α*, which is beneficial to fracture healing. We confirmed that miR-155 was upregulated or HIF-1*α* was downregulated, and the HIF-1*α* expression, VEGF, and Col-I was inhibited, which suggested that it affects angiogenesis and wound healing.

## 5. Conclusion

Diabetic foot ulcers are among the serious complications which are closely linked to diabetes mellitus. However, there is still a lack of accurate and effective standard prevention and treatment programs for DFU. In this manuscript, we have investigated the function of lncRNA CASC2/miR-155/HIF-1*α* in the wound healing of DFU. We have analyzed lncRNA CASC2's expression in the marginal tissues of ulcers in patients and mice with DFU. Additionally, the interaction relationship and mechanism between lncRNA CASC2, miR-155, and HIF-1*α* were determined, which proved the effects of lncRNA CASC2/miR-155/HIF-1*α* on fibroblasts apoptosis, proliferation, and migration. According to our study, the lncRNA CASC2's expression was low in the tissues of ulcers of DFU mice and patients. LncRNA CASC2's overexpression promoted fibroblasts migration, proliferation, and inhibited apoptosis and was beneficial for the healing of wounds, preferably in the DFU mice. In addition, lncRNA CASC2 directly targets miR-155 and HIF-1*α* functions as miR-155's target gene. Overexpression of miR-155 abrogated the function of lncRNA CASC2. Similarly, HIF-1*α*'s inhibition has reversed the effect of miR-155 downregulation on fibroblasts. In general, overexpression of lncRNA CASC2 facilitated wound healing through miR-155/HIF-1*α* in DFU. This provides a new strategy for the treatment of DFU.

## Figures and Tables

**Figure 1:** LncRNA CASC2 expression's downregulation and miR-155 expression's upregulation in DFU patients are as follows. (a) RT-qPCR detection of miR-155 expression in ulcer marginal tissues of DFU patients and foot tissues (preferably normal) of healthy individuals. (b) RT-qPCR detection of miR-155 expression in the marginal ulcer tissues of DFU patients and foot tissues (preferably normal) of healthy individuals. (c) Analysis of the expression's correlations of lncRNA CASC2 and miR-155 in ulcer tissues. ^*∗∗*^*p* < 0.01 vs. the control group.

**Figure 2:** Increased expression of lncRNA CASC2 contributes to DFU wound healing as follows. (a) RT-qPCR to reveal the level of expression of the lncRNA CASC2 in cells. (b, c) Cytometry of flow to evaluate the apoptosis of fibroblasts. (d) Wound healing assay to determine the change in migration ability of cells. (e) The proliferation activity of fibroblasts was measured by MTT. (f) Images of wound healing on the foot of DFU mice. (g) RT-qPCR to reveal the level of expression of lncRNA CASC2 in DFU mice. (h) Western blot was utilized for the measurement of the HIF-1*α*'s expression, VEGF, and Col-I in DFU mice. ^*∗∗*^*p* < 0.01, ^*∗*^*p* < 0.05, and ^*∗∗∗*^*p* < 0.001 against a group of DFU.

**Figure 3:** LncRNA CASC2 directly targeting miR-155. (a) Sequence alignment of the binding site between lncRNA CASC2 and miR-155. (b) The experiment of the dual-luciferase reporter gene detected the fluorescence activity of lncRNA CASC2-wt/mut under the treatment of miR-155/NC mimics, ^*∗∗*^*p* < 0.01 vs. group of CASC2-wt + NC mimics. (c) The lncRNA CASC2 expression, preferably after miR-155 mimics/inhibitor transfection, was performed by RT-qPCR, ^*∗∗∗*^*p* < 0.001 against a group of NC mimics and ^##^*p* < 0.01 against a group of NC inhibitor.

**Figure 4:** Overexpression of miR-155 abrogated the function of lncRNA CASC2. (a) Relative expression of lncRNA CASC2 was detected by RT-qPCR. (b, c), Flow cytometry to evaluate the apoptosis of fibroblasts. (d) The proliferation activity of the cell was measured by MTT. (e) Healing of wound assay to determine the ability of cells migration at 0 h and 24 h. (f) Western blot measurement of HIF-1*α*, VEGF, and Col-I protein expression levels in fibroblasts. ^*∗∗∗*^*p* < 0.001 and ^*∗∗*^*p* < 0.001 vs. group of DFU, ^#^*p* < 0.05, ^###^*p* < 0.001, and ^##^*p* < 0.01 against a group of DFU + CASC2.

**Figure 5:** HIF-1*α* was identified as a target miR-155 gene as follows. (a) Sequence alignment of binding site between HIF-1*α* and miR-155. (b) The experiments of the dual-luciferase reporter gene detected the fluorescence activity of HIF-1*α*-wt/mut under the treatment of miR-155/NC mimics, ^*∗∗∗*^*p* < 0.001 against a mimic group of HIF-1*α*-wt + NC. (c) Western blot measured the protein expression of HIF-1*α* level. (d) The expression of mRNA of HIF-1*α* after transfection of miR-155 mimics/inhibitor was performed by RT-qPCR. ^*∗∗*^*p* < 0.001 against a group of NC mimics and a group of NC inhibitor vs. ^##^*p* < 0.01.

**Figure 6:** Inhibition of HIF-1*α* overturned the effect of miR-155 downregulation on fibroblasts. (a) The relative miR-155's expression and HIF-1*α* were detected by RT-qPCR. (b, c) Flow cytometry to evaluate the apoptosis of fibroblasts. (d) The proliferation activity of the cell was measured by MTT. (e) Healing of wound assay to determine the cell's ability of migration at 0 h and 24 h. (f) The gel and histogram of HIF-1*α*, VEGF, and Col-I proteins in fibroblasts were detected by Western blot. ^*∗∗∗*^*p* < 0.001 and ^*∗∗*^*p* < 0.001 against group of DFU, ^##^*p* < 0.01^#^*p* < 0.05, and ^###^*p* < 0.001 against a group of DFU + si-miR-155.

## Data Availability

The datasets used and analyzed during the current study are available from the corresponding author upon reasonable request.
